RETRACTED

# The MicroRNA-217 Functions as a Potential Tumor Suppressor in Gastric Cancer by Targeting GPC5

**DOI:** 10.1371/journal.pone.0125474

**Published:** 2015-06-22

**Authors:** Hui Wang, Xiaolin Dong, Xin Gu, Rong Qin, Hongping Jia, Jianpeng Gao

**Affiliations:** 1 Department of Gastroenterology, The Affiliated YanAn Hospital of Kunming Medical University, Kunming, 650051, Yunnan, China; 2 Department of neurology, The Affiliated YanAn Hospital of Kunming Medical University, Kunming, 650051, Yunnan, China; 3 Department of General Surgery, The Affiliated YanAn Hospital of Kunming Medical University, Kunming, 650051, Yunnan, China; Sun Yat-sen University Medical School, CHINA

## Abstract

Gastric cancer (GC) is one of the most common malignancies worldwide. Emerging evidence has shown that aberrant expression of microRNAs (miRNAs) plays important roles in cancer progression. However, little is known about the potential role of miR-217 in GC. In this study, we investigated the role of miR-217 on GC cell proliferation and invasion. The expression of miR-217 was down-regulated in GC cells and human GC tissues. Enforced expression of miR-217 inhibited GC cells proliferation and invasion. Moreover, Glypican-5 (GPC5), a new ocncogene, was identified as the potential target of miR-217. In addition, overexpression of miR-217 impaired GPC5-induced promotion of proliferation and invasion in GC cells. In conclusion, these findings revealed that miR-217 functioned as a tumor suppressor and inhibited the proliferation and invasion of GC cells by targeting GPC5, which might consequently serve as a therapeutic target for GC patients.

## Introduction

Gastric cancer (GC) is the fourth most common human malignancies and the second leading cause of cancer-related deaths worldwide, with estimated one million new cases per year[1–4]. Despite recent advances in diagnostic method, surgical technique and new chemotherapy regimens, the long-term survival rate for GC is still quite low[5, 6]. In many patients, GC is diagnosed at advanced stage with extensive invasion and lymphatic metastasis. Successful therapeutic strategies are limited and the mortality is high[7]. Therefore, it is urgent to investigate the fundamental molecular mechanisms underlying the drug resistance, histological heterogeneity, and development of metastasis to identify novel markers for the diagnosis and treatment for GC.

MicroRNAs (miRNAs) are small, approximately 22-nucleotide, non-coding RNAs that function as negative regulators of protein coding genes at the posttranscriptional level[8, 9]. By binding to the complementary sequences in the 3’-untranslated regions (3’-UTR) of their target mRNAs, miRNAs can induce direct mRNA degradation or translational inhibition[10–13]. Increasing evidence has indicated that miRNAs are involved in many important biological processes, including cell proliferation, differentiation, apoptosis, angiogenesis and immune response. Deregulation of miRNAs may lead to aberrant gene expression in various diseases including gastric cancer[14–16]. However, the understanding of the role and function of miRNAs in the GC is still in the early stage. Likewise, the roles of many other aberrantly expressed miRNAs in GC development are still unknown.

RETRACTED

Downregulation of miR-217 is a frequent event in various cancers, suggesting its important role in tumorigenesis[17–19]. However, little is known about the potential role of miR-217 in GC. In this study, the expression of miR-217 was decreased in GC cell lines and tissues. In addition, lower expression of miR-217was associated with pTNM stage. Overexpression of miR-217 suppressed GC cell invasion and proliferation. Furthermore, luciferase reporter assay and western blot confirmed that miR-217might function as a tumor suppressor in GC by targetingGlypican-5(GPC5).

## Materials and Methods

### Ethics Statement

All patients agreed to participate in the study and gave written informed consent. This study and consent was approved by the ethical board of the institute of The Affiliated YanAn Hospital of Kunming Medical University and complied with Declaration of Helsinki.

### Tissue samples

Samples of human GC tissues and paired-adjacent non-tumor gastric tissues that were farther than 5 cm from the tumors were obtained from 50 patients who underwent surgery resection at the The Affiliated YanAn Hospital of Kunming Medical University. Fresh samples were snap frozen inliquid nitrogen immediately after resection and stored at -80°C. All samples were obtained with patients’ informed consent and were histological confirmed by staining with hematoxylin–eosin. The histological grade of cancers was assessed according to criteria set by the World Health Organization. None of the patients received radiotherapy or chemotherapy before surgery. The characteristics of patients are described in S1 Table.

### Cell lines and cell culture

Human gastric cancer cell lines SGC-7901, HGC-27, MGC-803, MKN-45 and one normal gastric epithelial cell line GES-1 (as control) were purchased from the Institute of Biochemistry and Cell Biology at the Chinese Academy of Sciences(Shanghai, China). SGC-7901, HGC-27, MGC-803, MKN-45 were propagated in RPMI 1640 medium (Invitrogen, Carlsbad, CA, USA)and GES-1 was propagated in Dulbecco’s modified Eagle’s medium (Invitrogen). All the media were supplemented with10% fetal bovine serum. Cell lines were cultured at 37°C in a humidified incubator of 5% CO2.

RETRACTED

### RNA extraction and qRT-PCR

Total RNA was extracted from frozen specimens (or the cells) using Trizol (Invitrogen) following the manufacturer’s guide. 1mL of RNA was used to measure the expression of miR-217 by quantitative RT-PCR (qRT-PCR) with the TaqMan miRNA reverse transcription kit andtheTaqMan miRNA assay-specific RT primers for miR-217 according to the instructions of the manufacturer (Applied Biosystems, Foster City, CA). The expression of U6 was used as internal control. Real-time PCR was performed with 1mL of each cDNA on a Step One Plus Real-Time PCR System (Applied Biosystems, Foster City, CA) in duplicates. The expression of miR-217 was defined based on the threshold cycle (Ct), and relative expression levels were calculated as22^-[(Ct of miR-217)-(Ct of U6)]^ after normalization with reference to expression of U6 small nuclear RNA[20, 21] (S2 Table).

### Western blot

Total protein was extracted from frozen specimens (or the cells) using a Total Protein Extraction Kit (KeyGen, Nanjing, China) according to the manufacturer’s instructions. Measurement of protein concentration was done using a BCA Protein Assay Kit (KeyGen). Western blot analysis was performed as previously described[22]. The primary antibodies used for western blot were rabbit polyclonal anti-GPC5(Santa Cruz Biotechnology, Santa Cruz, CA, USA), mouse monoclonal anti-GAPDH(Cell Signaling Technology, Beverly, MA, USA).

### Cell transfection

The miR-217 mimic, mimic control (scramble), miR-217 inhibitor, inhibitor control, pEZ-GPC5 and control vector were purchased from RiboBio (Guangzhou, China). The HGC-27 cells were seeded in six-well plates at 30% confluence one day prior to transfection. Lipofectamine2000 (Invitrogen) was used for transfection of plasmid alone or together with RNA oligonucleotides.

### Luciferase assays

cells of 8×10^3^ were plated into 96-well plates. After 24-hincubation, a mixture of 100-ng pLUC-3’-UTR, 5-pmol negative control, miR-217mimic was cotransfected with 20 ng Renilla into cells using Lipofectamine 2000. Twenty four hoursafter transfection, firefly and Renilla luciferase activities were measured with a Dual-Luciferase Reporter System (Promega, Madison, WI, USA). The transfection efficiency was normalized by cotransfection with a Renilla reporter vector.

### Cell proliferation

Cells (3,000/well) were collected and seeded in 96-wellplates and incubated at 37°C after transfection. After incubation for 1 to 5 days, to the media of each well was added 10% Cell Counting Kit-8 (CCK-8; Dojindo, Kumamoto,Japan), and the plates were further incubated for another 3 hours at 37°C. Then, the media was replaced with 150 mL dimethyl sulfoxide(DMSO; Sigma-Aldrich), and the absorbance was measured at 450 nm using a microplate reader (Sunrise). The assay was repeated 3 times with six replicates.

RETRACTED

### Northern blot

Total RNA was isolated from each tissue using TRIzol reagent (Invitrogen Life Technologies) and Northern blotting was conducted as previous described[23]. Following Perfect Hyb Plus hybridization at 68°C, membranes were developed and analyzed. Northern blots hybridized with an 18S ribosomal RNA (rRNA) cDNA were used as controls.

### Cell invasion

Invasion assays were performed in triplicate using Transwell invasion chambers coated with Matrigel (BD, USA) as described in the manufacturer’s protocol. Cells were transfected withmiR-217 mimics, inhibitor or negative control oligonucleotide, cultured for 48 h, and transferred on the top of Matrigel-coated invasion chambers in a serum-free DMEM (1 ×10^5^ cells per Transwell). DMEM containing 10% fetal calf serum was added to the lower chambers. After incubation for 24 h, cells that remained on the top of the filter were scrubbed off and cells that migrated to the lower surface were fixed in90% alcohol and followed by crystal violet stain.

### Histology

Histological diagnosis was according to the triple-site gastric biopsy method. Tissues were fixed overnight in buffered formalin, embedded in paraffin, cut to 3-μm thickness, and stained with hematoxylin-eosin (H&E) staining.

### Statistical analysis

Statistical analyses were performed using the SPSS 17.0 statistical software package. Experiments were repeated independently at least three times, and data presented as means ± SD. The association between miR-217 and GPC5 was analyzed using Spearman’s correlation test. Comparisons between groups for statistical significance were conducted with Student’s paired two tailed t-test or One-way ANOVA. P < 0.05 was considered as statistically significant.

## Result

### The expression of miR-217 is downregulated in GC cell lines

We firstly quantified the expression level of miR-217 in four human GC cell lines (SGC-7901, HGC-27, MGC-803, MKN-45) and GES-1 using northern blot (Fig 1A). The expression level of miR-217 wasdecreased in GC cell lines compared with GES-1. QuantitativeRT-PCR also showed that the expression of miR-217 was decreased in GC cell lines (SGC-7901, HGC-27, MGC-803, MKN-45) compared with GES-1, a normal gastric epithelial cell line(Fig 1B).

**Fig 1:** The expression of miR-217 is downregulated in GC cell lines. (A) The expression level of miR-217 in four human GC cell lines (SGC-7901, HGC-27, MGC-803, MKN-45) and GES-1 was quantified using Northern blot.(B) The expression of miR-217 was assessing in GC cell lines (SGC-7901, HGC-27, MGC-803, MKN-45)andGES-1using Quantitative RT–PCR.

RETRACTED

### MiR-217 is downregulated in GC tissues

Quantitative RT-PCR was used to examine miR-217 expression in 50 GC tissues and their paired adjacent noncancerous tissues. The representative histological characteristics of GC and its paired adjacent noncancerous tissues were shown in Fig 2A. Among 50 tumor tissues, 44 cases exhibited decreased miR-217 expression compared with the adjacent normal tissues (88%, 44 of 50, Fig 2B). The expression of miR-217 was lower in GC tissues than in adjacent noncancerous tissues (Fig 2C). Moreover, lower levels of miR-217 expression associated with the pTNM stage of GC patients (Fig 2D).

**Fig 2:** MiR-217 is downregulated in GC tissues. (A) The tissues were histological confirmed using H&E staining. (Original magnification, ×100). (B) miR-217 was detected in 50 GC patients by real-time PCR. Data are presented as log 2 T/N of fold change of GC tissues relative to non-tumor adjacent tissues. (C) The expression of miR-217 in GC tissues compared with normal tissues. The expression of miR-217 was normalized to U6 snRNA. (D) The statistical analysis of the association between miRNA level and pTNM stage (I, II, III and IV). *p<0.05, and **p<0.01, ***p<0.001. One-way ANOVA was performed for analysis.

### miR-217 inhibits GC cell proliferation and invasion

The expression of miR-217was increased in transfected HGC-27 cells using miR-217 mimics (Fig 3A) and decreased using miR-217 inhibitor (Fig 3B). The proliferation was reduced in the HGC-27 cells transfected withmiR-217 mimics compared with cells transfected with scramble or untreated (Fig 3C). Meanwhile, the proliferation was increased in HGC-27 cells transfected withmiR-217inhibitor compared with cells transfected with control or untreated (Fig 3D). The invasiveness of cells transfected with miR-217 mimics was decreased compared with the scramble group or control group cells and miR-217 inhibitor increased cell invasion compared with the scramble group or control group cells (Fig 3E).

**Fig 3:** miR-217 inhibits GC cell proliferation and invasion. (A) Real-time RT-PCR analysis of miR-217 in HGC-27 cells upon transfection ofmiR-217 mimic. The expression of miR-217 in HGC-27 cells transfected with miR-217 mimics was up-regulated.U6 snRNA was used as internal control. (B) The expression of miR-217 in HGC-27 cells transfected with miR-217inhibitor was down-regulated.U6 snRNA was used as internal control. (C) Ectopic miR‑217 expression significantly inhibited cell proliferation, as demonstrated by CCK8 assay. (D) Inhibition of miR-217 expression significantly promoted cell proliferation, as demonstrated by CCK8 assay. (E) Invasion analysis of HGC-27cells after treatment withmiR-217 mimics, inhibitors or scramble or control; the relative ratio of invasive cells per field is shown below, *p<0.05, ** p<0.01, and ***p<0.001.

RETRACTED

### miR-217 posttranscriptional reduces GPC5 expression by directly targeting its 3’UTR

Analysis using available algorithms indicated that GPC5 was a theoretical target gene of miR-217 (Fig 4A) [24]. To prove that miR-217 directly targeted the GPC53’UTR, we performed luciferase reporter gene assays. Ectopic of miR-217 reduced luciferase activity in the GPC5 wild-type reporter gene but not the mutant GPC5 3’UTR, indicating that miR-217 directly targeted the GPC5 3’UTR (Fig 4B). The mRNA level of GPC5 was decreased after transfection with miR-217 mimics and increased after transfection with miR-217 inhibitor using qRT-PCR (Fig 4C). Consistent with this result, the ability of miR-217 to regulate the expression of the GPC5 protein was verified by western blotting (Fig 4D).

**Fig 4:** miR-217 posttranscriptional reduces GPC5 expression by directly targeting its 3’UTR. (A) The 3'-UTR of GPC5 mRNA contains the binding sequences of miR-217. (B) Relative luciferase activity of the indicated GPC5reporter construct in HGC-27cells is shown. Firefly luciferase values were normalized to Renilla luciferase activity and plotted as relative luciferase activity. (C) miR-217 overexpression significantly reduced the GPC5 mRNA levels in the HGC-27 cells and miR-217 inhibitor significantly enhanced the GPC5 mRNA levels in the HGC-27 cells. (D) Western blotting was performed to examine the effects of miR-217 on the expression of GPC5. GAPDH was also detected as a loading control.

### Restoration of miR-217 inhibits GPC5-mediated GC cell proliferation and invasion

Overexpression of GPC5 promoted the GC cell proliferation and invasion. When miR-217 mimic and pEZ-GPC5 were cotransfected into HGC-27 cells, miR-217 expression reduced the GPC5-induced GC cell proliferation and invasion (Fig 5A and 5C). Inhibition of GPC5 reduced the GC cell proliferation and invasion. When miR-217 inhibitor and shGPC5 were cotransfected into HGC-27 cells, miR-217 inhibitor promoted the shGPC5-inhibited cell proliferation and invasion (Fig 5B and 5D).

**Fig 5:** Restoration of miR-217 inhibits GPC5-mediated GC cell proliferation and invasion. (A) The cell growth in HGC-27co-transfected with either miR-217 mimic or 2.0 μg pEZ-GPC5 or pCDNA empty vector using CCK-8 proliferation assay.(B) The cell growth in HGC-27co-transfected with either miR-217 inhibitor or 2.0 μg shGPC5 (knocks down GPC5) or pCDNA empty vector using CCK-8 proliferation assay.(C) The cell invasive in HGC-27co-transfected with either miR-217 mimic or 2.0 μg pEZ-GPC5 or pCDNA empty vector using invasion assay.(D) The cell invasive in HGC-27co-transfected with either miR-217inhibitor or 2.0 μg shGPC5 or pCDNA empty vector using invasion assay. *p<0.05, ** p<0.01, and ***p<0.001.

RETRACTED

### GPC5 is upregulated in GC cell lines and specimens

The expression of GPC5 was higher in GC cell lines (SGC-7901, HGC-27, MGC-803, MKN-45) compared with GES-1, a normal gastric epithelial cell line (Fig 6A). The protein levels of GPC5 were also higher in GC tissues than that in adjacent noncancerous tissues using western blot (Fig 6B).

**Fig 6:** GPC5 is upregulated in GC cell lines and specimens. (A) The mRNA expression of CPG5 was assessing in GC cell lines (SGC-7901, HGC-27, MGC-803, MKN-45) and GES-1 using Quantitative RT–PCR. (B) The protein level of CPG5 in eight human GC tissues and its adjacent normal controls was quantified using western blot.

## Discussion

GC causes nearly one million deaths worldwide per year[25]. Recently, accumulating evidence has suggested that miRNAs play a crucial role in the pathogenesis of GC through regulating cell proliferation, apoptosis, migration, ads invasion[26–28]. In this study, miR-217 was frequently downregulated in human GC cell lines and tissues and the lower level of miR-217 was associated with pTNM stage of GC. Further experiments indicated that overexpression of miR-217 can suppress GC cell migration and invasion. GPC5 was identified as a direct and functional target of miR-217. We conclude that miR-217 appears to be a novel tumor suppressor in GC and that downregulated miR-217 may contribute to tumor development and progression in GC patients. Downregulation of miR-217 is a frequent event in various cancers, suggesting its important role in tumorigenesis[17–19]. Li and his colleagues showed that miR-217 was down-regulated in clear cell renal cell carcinoma (ccRCC) compared to paired normal tissue[29]. Lower miR-217 expression level was associated with higher tumor grade and stage. In this study, miR-217 was frequently downregulated in GC. Intriguingly, patients with lower expression of miR-217 tended to have more advanced TNM stage, suggesting that low expression ofmiR-217was associated with GC progression. Further studies demonstrated that overexpression of miR-217 suppressed GC cell invasion and proliferation. Together with previous results, these data suggest that miR-217might play a crucial role in GC tissue homeostasis and deregulatedmiR-217 might contribute to the development of a stomach neoplasia.

To investigate the molecular mechanism of the tumor suppressor role of miR-217 in GC, we used luciferase reporter assay and western blot to confirm that GPC5 was a target of miR-217 in GC cells. To confirm the direct regulation of GPC5 by miR-217, we used GPC 3’ UTR reporter vector bearing the potential miR-217 binding site in the fluorescent reporter. Furthermore, qRT-PCR and western blot assay showed that overexpression of miR-217 inhibited GPC expression. Glypicans are a family of proteoglycans that are linked to the exocytoplasmic surface of the plasma membrane via a glycosyl phosphatidylinositol anchor[30, 31]. Six glypicans have been identified in mammals (GPC1 to GPC6)[32, 33]. GPC5 is mainly expressed in developing central nervous system, limbs, kidney, lung and liver[34, 35]. Recent studies have indicated that some GPCs, especially GPC3 andGPC5, might play an important role in regulating cancer progression[35, 36]. For example, *Zhang* et al. showed that GPC5 was highly expressed in SACC-M(high lung-metastatic cell line) and in clinical samples of salivary adenoid cystic carcinoma (SACC) cases with lung metastasis[36]. The overall expression level of GPC5 in clinical cases of SACC with lung metastasis was higher. Williamson et al. showed that the gene encoding GPC5was amplified in 20% of patients with alveolar rhabdomyosarcoma (RMS) and that this glypican was overexpressed in RMS patients. Moreover, down-regulation of GPC5 expression by siRNA inhibited the proliferation rate of RMS cells. Another study found that high levels of GPC5 expression predicted poor postsurgical survival times for curatively respected NSCLC patients, suggesting the value of GPC5 as a molecular prognostic indicator[35, 37]. In our study, the expression of GPC5 was higher in GC cell lines and the protein levels of GPC5 were also higher in GC tissues than in adjacent noncancerous tissues. Inhibition of GPC5 reduced the GC cell proliferation and invasion. Restoration of miR-217 inhibited GPC5-mediated GC cell proliferation and invasion. These results demonstrated that miR-217might act as a tumor suppressor in gastric cancer by targeting GPC5.

RETRACTED

In conclusion, the present study demonstrated that miR‑217was downregulated in GC tissues and cell lines. Low levels of miR-217 expression were associated with pTNM stage of patients. Ectopic miR‑217 expression resulted in inhibition of GC cell proliferation and invasion. Further investigation revealed that GPC5 was a potential target of miR‑217. miR‑217 may serve as a predictor for prognosis and a therapeutic target for GC patients.

## Supporting Information

S1 Table Summary of clinicopathological parameters of patients with gastric cancer. (DOCX)

S2 Table Primer sequence. (DOCX)
